The article "Three-Dimensional Skin CT Based on Intelligent Algorithm in the Analysis of Skin Lesion Sites Features in Children with Psoriasis" was retracted in 2023. Reasons: signs of a paper mill; compromised peer review; unreliable results or conclusions.

# Three-Dimensional Skin CT Based on Intelligent Algorithm in the Analysis of Skin Lesion Sites Features in Children with Psoriasis

**DOI:** 10.1155/2022/8195243

**Published:** 2022-01-28

**Authors:** Lina Wang, Youning Zheng, Ran Zhou, Wenfang Liu

**Affiliations:** ^1^Department of Dermatology, Hanzhong People's Hospital, Hanzhong, 723000 Shaanxi, China; ^2^Department of Pediatrics, Hebei General Hospital, Shijiazhuang, 050051 Hebei, China; ^3^Surgery Teaching and Research Office, Cangzhou Medical College, Cangzhou, 061001 Hebei, China

## Abstract

This research was to explore the application value of three-dimensional computed tomography (CT) based on artificial intelligent algorithm in analyzing the characteristics of skin lesions in children with psoriasis. In this study, 15 children with psoriasis were selected as the observation group, and 15 children with other skin diseases were selected as the control group. The CT images were optimized, and the feature selection was carried out based on artificial intelligent algorithm. Firstly, the results were compared with the results of simple skin three-dimensional CT to determine the effectiveness. Then, the two groups of three-dimensional skin CT image features of skin psoriasis-like hyperplasia, Munro microabscess, dermal papillary vascular dilation, and squamous epithelium based on intelligent algorithms were compared. After comparison, the detection rate of psoriasis-like hyperplasia, Munro microabscess, dermal papillary vascular dilation, and squamous epithelium in the observation group was higher than that in the control group, with significant difference and statistical significance (*P* < 0.05). In addition, the sensitivity of psoriasis-like hyperplasia, Munro microabscess, dermal papilla vascular dilatation, and squamous epithelium in children with psoriasis was 80.0%, 86.7%, 80.0%, and 93.3%, respectively. The specificity of psoriasis-like hyperplasia, Munro microabscess, dermal papilla vascular dilatation, and squamous epithelium in children with psoriasis was 86.7%, 93.3%, 60.0%, and 73.3%, respectively. The results showed that Munro microabscess and psoriasis-like hyperplasia had high sensitivity and specificity in all diagnostic items, which could be used as important features of skin lesion sites in the diagnosis of psoriasis in children. The research provides a basis for the clinical diagnosis of psoriasis in children, which is worthy of clinical promotion.

## 1. Introduction

Psoriasis is characterized by a layer of easily exfoliated silver-white scales on the skin erythema, which is called “Bai Bi” in traditional Chinese medicine. Because its name is easily confused with “psoriasis” (neurodermatitis) in traditional Chinese medicine and is inconsistent with the actual disease, it is renamed “psoriasis.” Psoriasis has the characteristics of long course, easy recurrence, and difficult to cure, repeatedly, which causes pain to patients [1, 2]. The etiology of psoriasis has not yet been clearly studied, and many mechanisms are still being explored. At present, it is believed that the etiology of psoriasis is not a single factor but is caused by a variety of factors. The currently determined pathogenic factors include heredity, infection, immune abnormalities, endocrine abnormalities, mental abnormalities, tobacco, alcohol, and drugs [3–5]. At present, the treatment of psoriasis is mainly based on the combination of internal and external drugs, which is also treated by certain physical therapy, such as ultraviolet therapy, photochemotherapy, and hydrotherapy [6]. Due to the long and recurrent course of the disease, it is difficult to adopt all treatment methods continuously for a long time. In order to prevent the toxic and side effects of drugs as well as drug resistance of the body, the main treatment methods include combination medication, alternate medication, and intermittent therapy [7, 8]. In recent years, the national coordination conference on the prevention and treatment of psoriasis has proposed that the hormone drugs and hormone anticancer drugs used in recent years have a certain effect on psoriasis, but more serious side effects are caused, and integrated traditional Chinese medicine and Western medicine are the best means for the treatment of psoriasis. Therefore, a diagnostic method is urgently needed to assist treatment [9–11].

Currently, psoriasis is mainly diagnosed by skin computed tomography- (CT-) confocal laser scanning microscopy (CLSM), dermatoscopy examination, blood examination, skin biopsy, and trace element examination [12–14]. Due to the effectiveness and convenience of examination, skin CT examination has become the most widely used detection method. Compared with dermatoscopy examination, it can show the structural characteristics of subcutaneous tissue lesions in detail. Compared with other examination methods, it is convenient and fast and suitable for clinical promotion [15–17].

In recent years, with the development of computer-aided diagnosis (CAD) technology, the accuracy of diagnosis technology has made great progress by upgrading the traditional imaging technology. Dash et al. [18] pointed out that the application of various artificial intelligence algorithms made imaging diagnosis adapt to the diagnosis requirements of different skin diseases. For this study, the combination of artificial intelligent algorithm and feature analysis of CT images can effectively improve the deep learning of diagnostic features, so as to quickly and accurately annotate the feature tissue parts in a large number of images. Therefore, the combination of 2-3-dimensional hybrid convolutional neural network-based automatic segmentation algorithm and CT image will have a good application prospect in the feature analysis of psoriasis lesions sites [19, 20].

In order to improve the accuracy and efficiency of clinical diagnosis of pediatric psoriasis, three-dimensional skin CT based on artificial intelligent algorithm was innovatively applied to analyze the characteristics of skin lesions sites in children. In this study, 15 children with psoriasis in hospital were selected as the observation object, and 15 children with other skin diseases were selected as the control group. Moreover, CT image feature analysis based on artificial intelligence algorithm was used to diagnose the patients. By comparing the diagnostic information of the two groups, the diagnostic function of CT image feature analysis in psoriasis skin lesions sites was judged.

## 2. Research Objects and Methods

### 2.1. Research Objects

In this study, 15 children with psoriasis diagnosed in hospital were collected as the observation group, including 8 males and 7 females aged from 6 to 12 years old, with an average age of 9.73 ± 2.24 years old, including 9 in progressive stage, 5 in stable stage, and 6 in regression stage. 15 children with other skin diseases were selected as the control group, including 8 males and 7 females, aged from 7 to 12 years, with an average age of 9.89 ± 2.14 years. There were 5 cases of pityriasis rosea, 5 cases of chronic eczema, 2 cases of lichen planus, 2 cases of seborrheic dermatitis, and 1 case of herpes zoster. This study was approved by the ethics committee of hospital. Patients and their families were aware of this study and signed informed consent.

Inclusion criteria are as follows: (1) no other skin diseases in children with psoriasis. (2) The selected age is not more than 12 years old.

Exclusion criteria are as follows: (1) family members and patients are unwilling to participate. (2) Children with poor dependence.

### 2.2. Research Scheme

Patients in both groups were examined by three-dimensional skin CT system. Appropriate postures should be selected for detection, and appropriate amount of tap water should be applied to the lesion. Three-dimensional skin CT examination should be carried out in the patient's affected area with B-ultrasound coupling agent as the medium, and the scanning area was 500 *μ*m × 500 *μ*m. Three-dimensional imaging such as psoriasis-like hyperplasia of skin, Munro microabscess, dermal papillary vascular dilation, and squamous epithelium should be judged. The results of the two groups were compared to determine the role of skin psoriasis-like hyperplasia, Munro microabscess, dermal papillary vascular dilation, and squamous epithelium in the diagnosis of psoriasis in children.

Diagnostic function will be judged by sensitivity and specificity, and the specific calculation method is as follows.

(1) $$\begin{array}{c} M=\frac{\text{TP}}{\text{TP}+\text{FN}}\times 100\%, \end{array}$$

(2) $$\begin{array}{c} T=\frac{\text{TN}}{\text{TN}+\text{FP}}\times 100\%, \end{array}$$

(3) $$\begin{array}{c} M=\frac{O}{O_{N}}, \end{array}$$

(4) $$\begin{array}{c} T=\frac{C}{C_{N}}. \end{array}$$

Equations (1) and (2) are general equations for calculating sensitivity and specificity, where *M* is sensitivity, *T* is specificity, TP is the number of true positive cases, FN is the number of false negative cases, TN is the number of true negative cases, and FP is the number of false positive cases. Equations (3) and (4) are the calculation equations used in this study, where *O* is the number of positive cases in the observation group, *O*_*N*_ is the total number of cases in the observation group, *C* is the number of positive cases in the control group, and *C*_*N*_ is the total number of cases in the control group.

### 2.3. Three-Dimensional Skin CT Based on Artificial Intelligence Algorithm

In this study, 2-3-dimensional hybrid convolutional neural network-based automatic segmentation algorithm is utilized to process CT images. First, the original images are preprocessed. According to pixel value-CT value conversion equation, the CT value of window range is calculated. *X* refers to pixel value, *S* denotes zoom ratio, and *P* represents deviation value. CT value is calculated by Equation (5).

(5) $$\begin{array}{c} CT=X\times S+P. \end{array}$$

Next, the images are truncated according to window range, and the truncated data *A* and *B* need to be calculated by deviation standardization Equation (6).

(6) $$\begin{array}{c} B=\frac{A-a^{\min}}{a^{\max}-a^{\min}}. \end{array}$$

After the preprocessing, other interference is eliminated and 2-3-dimensional hybrid network is utilized to segment images. The backbone network 2-dimensional component is ResNet34, and the backbone network 3-dimensional component uses ResNet18. ResNet is an excellent image classification and segmentation model, and the residual structure in the model makes it easier to be optimized. The residual structure can address the problem of the disappearance of propagation gradient caused by reverse propagation in the propagation of neural network. In addition, gradient information is propagated easier in reverse propagation process with the residual structure. The networks added into residual modules will obtain higher recognition accuracy.  Figure 1 shows the specific structure model of ResNet.

The specific segmentation process of 2-3-dimensional hybrid network-based segmentation algorithm consists mainly of the next several steps. Firstly, the preprocessed images are reorganized. Secondly, 2-dimensional network input is transmitted into 2-dimensional model for the completion of extraction of 2-dimensional segmentation results and 2-dimensional features. Thirdly, 2-dimensional segmentation results are converted into 3-dimensional forms. Next, 3-dimensional network original input is combined to complete 3-dimensionl network input. After that, 2-dimensional features are converted into 3-dimensional features, and then, 3-dimensional features and 3-dimensional network input are transmitted into 3-dimensional model simultaneously to obtain the 3-dimensional segmentation results. Finally, maximum connected domain processing is performed for the 3-dimensional segmentation results to obtain the final segmentation results.  Figure 2 displays the process framework.

The model is trained. The 2-dimensional network, the 3-dimensional network, and 2-3-dimensional hybrid network are trained separately. Cross entropy (*J*) is expressed by Equation (7).

(7) $$\begin{array}{c} J=\overset{x}{\underset{x_{i}=1}{\sum }}\left[b_{i}\log\overset{ˇ}{b_{i}}+\left(1-b_{i}\right)\left(1-\log\overset{ˇ}{b_{i}}\right)\right]. \end{array}$$

### 2.4. Statistical Research

In this study, SPSS 11.5 was used as the analysis and statistical software of data processing for *χ*^2^. *t*-test was used. It was expressed as mean ± standard deviation ($\overset{¯}{\text{x}}\pm \text{s}$), and *P* < 0.05 meant that the difference was statistically significant.

## 3. Results

### 3.1. Algorithm Simulation Results

Figure 3 shows the three-dimensional skin CT image of a 7-year-old patient with psoriasis.

The test image is divided into 8 × 8 image blocks, and Figure 3 is reconstructed. The results are as follows.

Figure 4(a) is a 2D reconstructed image.  Figure 4(b) is a reconstructed image of 3D.  Figure 4(c) is an image reconstructed by 2-3D algorithm. The artificial intelligence algorithm was used to optimize CT images, which can improve the appearance of small tissue cells in CT images and the contrast between characteristic lesions and ordinary cells. This experiment proved that the 2-3D algorithm was better than the original images and the commonly used 2D algorithm and 3D algorithm in improving image accuracy.

The comparison between the corresponding maximum value, minimum value, and average of 2D algorithm, 3D algorithm, and 2-3D algorithm is shown in Figure 5.

The comparison shows that the average value, the minimum value, and the maximum value of 2-3D hybrid intelligence algorithm are all significantly higher than those of 2D intelligence algorithm and 3D intelligence algorithm. Besides, the variance of 2-3D hybrid intelligence algorithm is obviously less than that of 2D intelligent algorithm and 3D intelligent algorithm, which demonstrates that 2-3D hybrid intelligence algorithm possesses more excellent performance with higher stability and reliability.

### 3.2. General Data Statistics

Figure 6 is gender comparison of two groups of children. In the observation group, 15 children with psoriasis were diagnosed, aged from 6 to 12 years, with an average age of 9.27 ± 1.83 years, including 8 males and 7 females. In the control group, 15 nonpsoriasis children were aged 7~12 years, with an average age of9.73 ± 1.62years. And there was no statistical significance in age and gender differences, which was comparable.

### 3.3. Characteristic Analysis of Psoriatic Lesions

Figure 7 is a three-dimensional CT image of the skin lesion sites of a child with herpes zoster.

As shown in Figure 7, there was no characteristic of psoriasis-like hyperplasia, Munro microabscess, dermal papillary vascular dilation, and squamous epithelium at the lesion site of herpes zoster. All diagnostic results are summarized, and the results are shown in Figure 8.

The two groups of data are summarized and calculated, respectively. The data and calculation results are shown in Table 1.

## 4. Discussion

Skin three-dimensional CT, also known as confocal laser scanning microscope (CLSM), is a new dermatological examination method to scan and image the skin lesion sites through the probe and observe the lesions at the cellular level. Compared with traditional dermatological examination methods, skin three-dimensional CT not only has the characteristics of simple operation, real-time fast, dynamic response, no wound, high repeatability, and simultaneous examination of multiple lesions but also plays a more and more important role in the daily examination and diagnosis of dermatology. Li et al. [21] also conducted in-depth research on the scope, accuracy, and specificity of skin three-dimensional CT in the diagnosis of various skin diseases. Firstly, the algorithm interpretation and verification experiments of CT image optimization based on artificial intelligence algorithm were carried out. In this experiment, the artificial intelligent algorithm was used to optimize the CT image, so as to improve the appearance of CT image on small tissues and cells and improve the contrast between characteristic lesions and general cells, so as to achieve feature analysis. Through verification experiments, it was confirmed that the artificial intelligent algorithm had better improvement in image accuracy than the original image and the commonly used K-SVD algorithm and SAE algorithm.

In this study, 15 children with psoriasis diagnosed in clinic were selected. 15 cases of other common skin diseases that are easily confused with psoriasis, such as pityriasis rosea, herpes zoster, and chronic eczema, were selected as the control group and compared with psoriasis patients. Both groups underwent CT images based on the above artificial intelligent algorithm. In the final results, 12 cases of psoriasis-like hyperplasia, 13 cases of Munro microabscess, 12 cases of dermal papilla vascular dilation, and 14 cases of squamous epithelium were detected in 15 children with psoriasis. In the control group, there were 2 cases of psoriasis-like hyperplasia, 1 case of Munro microabscess, 6 cases of dermal papilla vascular dilation, and 4 cases of squamous epithelium. The data of the two groups were statistically analyzed, and there were significant differences (*P* < 0.05). The sensitivity and specificity of psoriasis-like hyperplasia, Munro mircroabscess, dermal papilla vascular dilation, and squamous epithelium were calculated, and the sensitivity was 80.0%, 86.7%, 80.0%, and 93.3%, respectively. The specificity was 86.7%, 93.3%, 60%, and 73.3%, respectively. For the combination of sensitivity and specificity, it can be obviously found that the sensitivity and specificity of Munro microabscess were among the top, which was the best analysis feature of the lesions' parts of psoriasis skin. The comprehensive data of psoriasis-like hyperplasia were slightly lower than those of Munro microabscess, but also higher than those of squamous epithelium and dermal papilla vascular dilation.

In this study, it is determined that CT images based on intelligent algorithm play a positive role in the analysis of the characteristics of psoriasis in children, especially the examination of psoriasis-like hyperplasia, Munro microabscess, dermal papilla vascular dilation, and squamous epithelium. It is proved that these four types of features can be used as the diagnostic features of three-dimensional CT of psoriatic skin in children, especially Munro microabscess and psoriasis-like hyperplasia, which have high sensitivity and specificity, which is similar to the research results of Lv et al. [22].

Qing et al. [23] found that the main causes of psoriasis in children are infection and dietary metabolism. If there is a family genetic history, it will aggravate the condition of psoriasis. Žurauskas et al. [24] performed noninvasive optical examination on 33 patients with psoriasis, 7 patients with eczema, and 18 patients with healthy skin. An image data collection method based on fully automatic feature extraction algorithm was used to study the skin features of patients. The results showed that both eczema and psoriasis had inflammation. The degree of inflammation in eczema will be lower than that in psoriasis. For this verification, combined with the erythema, scale, and thickness of the lesion, this study proposes a marker score for the diagnosis of psoriasis. Errichetti and Stinco [25] studied the dermoscopic characteristics of psoriasis and chronic eczema. The results showed that diffuse white scales were very significant in psoriasis, while light yellow scales, brownish orange dots/balls, and yellowish orange scabs were found in chronic eczema. Shrivastava et al. [26] observed and summarized the characteristics of skin color and texture samples at 540 lesions of 30 Indian psoriasis patients and proposed a fully automatic algorithm for psoriasis feature diagnosis.

## 5. Conclusion

In this study, 15 children with psoriasis were selected as the observation object, and the characteristics of skin three-dimensional CT images based on artificial intelligence were analyzed and compared. The results show that the three-dimensional CT image of skin based on artificial intelligence has high sensitivity and specificity in four types of analysis features. It is proved that this detection method can be used in the clinical analysis of the characteristics of psoriasis in children and is worthy of popularization. Due to the small number of children with psoriasis and other skin diseases, this experiment cannot pass the validation experiment of a large amount of data. The experimental data may have some errors, but the results will not be too different. It is expected that relevant organizations or teams can select more patients for research in the future. In this study, the three-dimensional CT image of the skin is optimized to analyze the characteristics of the site of skin lesion, which provides certain research data and feature selection for the diagnosis of psoriasis in children and has certain significance for clinical experiment and diagnosis in the future.

## Figures and Tables

**Figure 1:** ResNet structure.

**Figure 2:** 2-3-dimensional segmentation algorithm process framework.

**Figure 3:** Three-dimensional CT of skin in patients with psoriasis (male, 7 years old, Munro microabscess). It is the conglomeration of large refractive particles, which have a flicker or flow feeling during dynamic scanning.

**Figure 4:** Reconstructed image results.

**Figure 5:** Comparison of 2D algorithm, 3D algorithm, and 2-3D algorithm [17]. Note: ∗ indicates that the difference is statistically significant compared with 2D and 3D, *P* < 0.05.

**Figure 6:** Gender comparison of two groups of children.

**Figure 7:** Three-dimensional CT of the skin lesion sites in children with herpes zoster.

**Figure 8:** Comparison of positive and negative characteristic observation results of the two groups: (a) the positive composition of the observation group, (b) the negative composition of the observation group, (c) the positive composition of the control group, and (d) the negative composition of the control group.

**Table 1:** Skin three-dimensional CT test results and calculation results of the observation group and the control group.

	Observation		Control		Sensitivity (%)	Specificity (%)	*P*
	Positive	Negative	Positive	Negative			
Psoriasis-like hyperplasia	12^∗^	3^∗^	2	13	80	86.7	<0.05
Munro microabscess	13^∗^	2^∗^	1	14	86.7	93.3	<0.05
Dermal papillary vascular dilation	12^∗^	3^∗^	6	9	80	60	<0.05
Squamous epithelium	14^∗^	1^∗^	4	11	93.3	73.3	<0.05

Note: ∗ indicates that the difference is statistically significant compared with the control group, *P* < 0.05.

## Data Availability

The data used to support the findings of this study are available from the corresponding author upon request.
